# Analysis of the Application Value of Echocardiography Combined with CK-MB, Alb, and CysC in the Prognosis Assessment of Patients with Chronic HF

**DOI:** 10.1155/2022/3986646

**Published:** 2022-08-30

**Authors:** Yiyi Ma, Dongxiao Zhu, Xinyan Chen, Baihong Li, Jun Zhu

**Affiliations:** ^1^Department of Ultrasound, Affiliated Hospital of Jiangnan University, Wuxi 214122, China; ^2^Internal Medicine-Cardiovascular Department, Affiliated Hospital of Jiangnan University, Wuxi 214122, China

## Abstract

In order to evaluate the diagnostic and prognostic value of echocardiography combined with serum creatine kinase-MB (CK-MB), albumin (Alb), and cystatin C (CysC) in patients with chronic heart failure (HF), 93 patients diagnosed with chronic HF in our hospital from March 2019 to January 2020 are retrospectively analyzed and included in the HF group. Another 100 healthy subjects who come to our hospital for general physical examination are selected as the control group. Echocardiography is used to detect the cardiac parameters of each group. The experimental results show that echocardiography parameters combined with CK-MB, Alb, and CysC have high application value in diagnosis and evaluation of patients with chronic HF, which can provide theoretical basis for improving the prognosis of patients with chronic HF through real-time monitoring of the above indicators.

## 1. Introduction

Heart failure (HF), as a kind of disease caused by myocardial injury, leads to changes in ventricular structure and function [1]. As a continuous state of HF, chronic HF is also one of the important causes of death [2]. According to global statistics, with the increasing aging population in China, the morbidity and mortality of chronic HF are also on the rise year by year, and the prognosis of most patients is poor, and the clinical symptoms, such as joint swelling, fatigue, and dyspnea, have a serious impact on the quality of life of patients [3, 4]. Therefore, it is of great significance to evaluate the prognosis of patients with chronic HF by highly accurate and sensitive prediction method to improve the prognostic survival rate and individual management level of this group [5]. Echocardiography has the characteristics of high safety and non-invasive, and has been praised by clinicians, but some scholars point out that a single ultrasonic echocardiography test cannot accurately reflect the changes of myocardial function, so it still needs other specific serum indexes for testing [6]. Studies have shown that creatine kinase-MB (CK-MB), as a marker of myocardial injury, can be upregulated when myocardial injury occurs. Cystatin C (CysC) also plays an important role in the pathogenesis of various vascular diseases. Albumin (Alb) is also considered to be an independent predictor of death and prognosis in patients with chronic HF. Therefore, in this study, 93 patients with chronic HF are selected to further analyze the differences in echocardiography parameters, CK-MB, Alb, and CysC expression, and to evaluate the clinical value of combined detection for diagnosis and prognosis, laying a theoretical foundation for improving the prognosis of patients with chronic HF.

The rest of this paper is organized as follows.  Section 2 discusses related work, followed by evaluating the clinical value of combined detection for diagnosis and prognosis in Section 3. The comparison of clinical data and result analysis is discussed in Section 4.  Section 5 concludes the paper with summary.

## 2. Related Work

As a common type of cardiovascular disease in clinical practice, the incidence of chronic HF [7–9] usually increases with the increase of age, and it is also one of the important causes of cardiovascular disease death in the elderly, seriously threatening people's life and health [10]. According to clinical studies, the pathological features of chronic HF are usually reflected in neuroendocrine disorders, myocardial remodeling, increased preload, and so on [11]. Therefore, a diagnosis and prediction method with high sensitivity and specificity is of great clinical significance for patients with chronic HF. Although multiple indicators are closely related to the development of chronic HF at present, it is susceptible to other factors and cannot be accurately diagnosed and predicted [12]. Echocardiography, as an imaging diagnosis method, commonly used to detect heart structure and function in clinical practice, plays an important role in the detection of various cardiovascular diseases [13].

When two indexes exceeded the normal value, left ventricular enlargement is considered, and heart function impairment should be warned at this time [14]. Left ventricular ejection fraction (LVEF) is an important indicator to evaluate left ventricular function. The lower the LVEF is, the more severely impaired the left ventricular function is. However, chronic HF patients are often accompanied by cardiovascular diseases such as history of heart disease, coronary heart disease, and hypertension, resulting in changes in cardiac structure and function, thus showing differences in echocardiographic parameters [15]. In addition, as a widely distributed serum marker of myocardial tissue, CK-MB has a very low serum content in normal people. When a large amount of CK-MB is released into the blood, CK-MB levels can be detected in the serum. With the aggravation of cardiomyocyte injury, the release level of CK-MB increased gradually. It is consistent with the results of this study [16]. Charokopos et al. [17] pointed out that the increase of Alb was closely related to the improvement of cardiac function, which indicated that Alb is normally secreted by the liver of the body, but for patients with chronic HF, the decrease of cardiac displacement leads to the decrease of liver blood perfusion, which leads to the increase of venous pressure and hinders venous blood return. Blood clots the liver cells and reduces Alb secretion. In addition, other scholars showed that decreased Alb level was also closely related to protein loss. According to their analysis, gastrointestinal tract congestion is caused by decreasing cardiac discharge in patients with chronic HF, which hinders the absorption of protein by the gastrointestinal tract, thus resulting in decreasing detectable Alb content in serum [18]. Moreover, CysC, as a cysteine protease inhibitor, can be produced by the body's tissues and organs more common. Also, by participating in the extracellular matrix remodeling, CysC can reduce collagen protein decomposition rate which is involved in the pathogenesis of chronic HF process. When the CysC level rises in patients with chronic HF, myocardial collagen decomposition rate is higher than synthetic rate [19].

## 3. Echocardiographic Examinations and Enzyme-Linked Immunosorbent Assay

### 3.1. General Information

A retrospective analysis is performed on 93 patients diagnosed with chronic HF in our hospital from March 2019 to January 2020, and they are included in the HF group. Another 100 healthy people who underwent general physical examination in our hospital are selected as the control group. In addition, patients in the chronic HF group are divided into good group (*n* = 42) and poor group (*n* = 51) according to different prognostic outcomes. The comparison of baseline data of each group is shown in Table 1, which is comparable (*P* > 0.05). The clinical data and general information collected in this study will only be used for clinical research and will not be used for other purposes.

Inclusion criteria were as follows: (1) meet the clinical diagnostic criteria for chronic HF; (2) complete clinical data and general information; (3) good communication skills and compliance; and (4) no record of loss to follow-up.

Exclusion criteria were as follows: (1) combined with mental system diseases; (2) congenital immune dysfunction; (3) complicated with heart, liver, kidney, and other major organ diseases, affecting the study indicators; and (4) poor research coordination.

### 3.2. Echocardiographic Examination

All subjects underwent color Doppler ultrasound examination (purchased from Dawei Medical Co. LTD. (Model: WD-F3)). Echocardiography was performed. During the examination, the probe is placed at the apex of the heart and beside the sternum in the left decubitus position. The depth, contrast, and enhancement are constantly adjusted to obtain clear images.

5 ml of fasting venous blood is taken from the subjects in the morning and put into a centrifuge with centrifugation parameters set at 3500 r/min and centrifugation radius of 12.5 cm for 10 min. Supernatant is retained for testing. Serum levels of CysC and CK-MB in each group are detected by enzyme-linked immunosorbent assay in strict accordance with the operating instructions. Both CysC and CK-MB kits are purchased from Shanghai Jingjing Antibiotics Co. LTD.

### 3.3. Observation Indicators

Observation indicators are as follows:

  (1) Comparison of echocardiography parameters and expression differences of CK-MB, Alb, and CysC between HF group and control group is conducted.
  (2) ROC curve is drawn to evaluate the diagnostic efficacy of echocardiography parameters combined with CK-MB, Alb, and CysC for chronic HF.
  (3) Comparison of echocardiography parameters and CK-MB, Alb, and CysC expressions between the good group and the bad group is conducted.
  (4) Kaplan–Meier survival curve is drawn to observe the effects of high and low expression of CK-MB, Alb, and CysC on the prognosis and survival rate of HF patients.
  (5) ROC curve is drawn to evaluate the predictive efficacy of echocardiography parameters combined with CK-MB, Alb, and CysC for the prognosis of patients with chronic HF.

### 3.4. Statistical Processing

SPSS 25.0 statistical software is used for data analysis:

  (1) Measurement data: if the data follow normal distribution and homogeneity of variance after normality test, they are represented by mean ± standard deviation. Paired sample *T* test is used for intra-group test, and variance comparison is used between groups.
  (2) Count data: descriptive statistical analysis is conducted by percentage, and *x*^2^ test is performed.
  (3) ROC curve is drawn to observe the evaluation value of echocardiography parameters combined with CK-MB, Alb, and CysC in diagnosis and prognosis of patients with chronic HF.
  (4) Kaplan–Meier survival curve observes the effects of high and low expression of CK-MB, Alb, and CysC on the prognosis and survival rate of HF patients. All the above data show significant differences with *P* < 0.05.

## 4. Clinical Data and Result Analysis

### 4.1. Comparison of Ultrasonic Cardiac Parameters and Expression Differences of CK-MB, Alb, and CysC

Table 2 shows the differences in echocardiography parameters and expression of CK-MB, Alb, and CysC. It is clearly evident from Table 2 that ultrasonic echocardiography parameters and laboratory test results show that LVEF and Alb in patients with chronic HF are significantly lower than those in the normal group, while left ventricular end-diastolic dimension (LVEDD), left ventricular end-systolic dimension (LVESD), CK-MB, and CysC are significantly higher than those in the normal group (all *P* < 0.05).

Table 3 shows the diagnostic efficacy of each indicator. It is clearly evident from Table 3 that LVEF is derived from (LVED-LVESD)/LVEDD, and only LVEF is included in the joint diagnosis.

Figure 1 shows the ROC chart of each indicator detection. It is clearly evident from Figure 1 that the area under the curve of the joint diagnosis is significantly higher than that of the single test.

### 4.2. Comparison of Echocardiography Parameters and CK-MB, Alb, and CysC Expressions

Table 4 shows the differences in echocardiography parameters and expression of CK-MB, Alb, and CysC. It is clearly evident from Table 4 that LVEF and Alb in the poor group are significantly lower than those in the good group, while LVEDD, LVESD, CK-MB, and CysC are significantly higher than those in the good group (all *P* < 0.05).

Figure 2 shows that the high expression and low expression of CK-MB affect prognosis and survival. It is clearly evident from Figure 2 that low expression of CK-MB is significantly higher than that of patients.

Figure 3 shows that the high expression and low expression of CysC affect prognosis and survival. It is clearly evident from Figure 3 that low expression of CysC is significantly higher than that of patients.

Figure 4 shows that the high expression and low expression of Alb affect prognosis and survival. It is clearly evident from Figure 4 that the 1-year survival rate of patients with high expression of Alb is higher than that of patients with low expression of Alb.

Table 5 shows the diagnostic efficiency of each index. It is clearly evident from Table 5 that in sensitivity analysis, the value of CysC is the smallest.

Figure 5 shows the ROC chart of each indicator detection. It is clearly evident from Figure 5 that the area under the curve of joint prediction is significantly higher than that of single detection.

Through the above experimental results, it can be observed that the LVEF and Alb of patients with chronic HF are significantly lower than those of the normal group, and LVEDD, LVESD, CK-MB, and CysC are significantly higher than those of the normal group (all *P* < 0.05). LVEF and Alb of patients with poor prognosis are lower than those of patients with good prognosis. At the same time, LVEDD, LVESD, CK-MB, and CysC are higher, which indicates that LVEDD is commonly used to evaluate left ventricular diastolic function in clinical work, while LVESD is used to evaluate left ventricular systolic function.

## 5. Conclusion

Echocardiography and serum CK-MB, CysC, and Alb expressions in patients with chronic HF are closely related to the degree of disease, and the prognosis of such patients can be accurately evaluated by real-time monitoring of the changes of each indicator, which is worthy of clinical application. In the future work, this study will analyze the role of combined detection in the diagnosis and prognosis assessment of patients with chronic HF by combining it with CK-MB, CysC, and Alb.

## Figures and Tables

**Figure 1:** ROC chart of each indicator detection.

**Figure 2:** High expression and low expression of CK-MB affect prognosis and survival.

**Figure 3:** High expression and low expression of CysC affect prognosis and survival.

**Figure 4:** High expression and low expression of Alb affect prognosis and survival.

**Figure 5:** ROC chart of each indicator detection.

**Table 1:** Baseline data.

	HF group (*n* = 93)	Control group (*n* = 100)	Good group (*n* = 42)	Bad group (*n* = 51)
Age (years)	52.92 ± 9.83	54.10 ± 9.22	51.76 ± 8.66	53.88 ± 10.68
Gender				
Male	46(49.46%)	55(55.00%)	24(57.14%)	22(43.14%)
Female	47(50.54%)	45(45.00%)	18(42.86%)	29(56.86%)
BMI (kg/m^2^)	25.11 ± 1.77	25.01 ± 1.86	24.81 ± 1.70	25.36 ± 1.80

**Table 2:** Differences in echocardiography parameters and expression of CK-MB, Alb, and CysC.

Group	*n*	CK-MB (IU/L)	Alb (g/L)	CysC (mg/L)	LVEF (%)	LVEDD (mm)	LVESD (mm)
HF group	93	50.05 ± 10.60	33.39 ± 2.21	4.32 ± 1.07	36.41 ± 4.97	63.61 ± 7.15	50.55 ± 4.25
Control group	100	9.08 ± 2.17	41.90 ± 2.06	0.64 ± 0.67	63.18 ± 7.60	44.22 ± 2.61	34.46 ± 5.42
*t*		37.819	−27.691	34.405	−28.731	25.367	22.837
*P*		＜0.001	＜0.001	＜0.001	＜0.001	＜0.001	＜0.001

**Table 3:** Diagnostic efficiency of each index.

	95% CI	Sensitivity (%)	Specificity (%)	AUC	Cutoff value
The joint detection	0.662∼0.858	76.50	79.30	0.782	—
LVEF	0.489∼0.716	69.20	65.70	0.602	50.00%
CK-MB	0.461∼0.689	64.20	61.20	0.575	21.34 IU/L
Alb	0.525∼0.747	51.80	61.50	0.636	36.62 g/L
CysC	0.448∼0.686	57.50	59.60	0.567	1.95 mg/L

**Table 4:** Differences in echocardiography parameters and expression of CK-MB, Alb, and CysC.

Group	*n*	CK-MB (IU/L)	Alb (g/L)	CysC (mg/L)	LVEF (%)	LVEDD (mm)	LVESD (mm)
Good group	42	39.95 ± 5.71	35.04 ± 1.71	3.43 ± 0.72	41.48 ± 2.10	56.95 ± 4.70	46.57 ± 1.63
Bad group	51	58.37 ± 4.86	32.03 ± 1.56	5.06 ± 0.67	32.24 ± 1.58	69.10 ± 2.83	53.82 ± 2.61
*t*		16.790	−8.834	11.313	−24.199	15.384	15.691
*P*		＜0.001	＜0.001	＜0.001	＜0.001	＜0.001	＜0.001

**Table 5:** Diagnostic efficiency of each index.

	95% CI	Sensitivity (%)	Specificity (%)	AUC	Cutoff value
The joint detection	0.764∼0.928	82.50	81.70	0.846	—
LVEF	0.593∼0.810	72.20	76.30	0.702	45.60%
CK-MB	0.485∼0.714	67.80	67.40	0.599	45.64IU/L
Alb	0.650∼0.850	69.70	74.20	0.750	34.24 g/L
CysC	0.530∼0.759	64.70	69.10	0.645	4.29 mg/L

## Data Availability

The simulation experiment data used to support the findings of this study are available from the corresponding author upon request.

## References

[1] Roger V. L. (2021). Epidemiology of heart failure: a contemporary perspective. *Circulation Research*.

[2] Pontremoli R., Borghi C., Perrone Filardi P. (2021). Renal protection in chronic heart failure: focus on sacubitril/valsartan. *European Heart Journal-Cardiovascular Pharmacotherapy*.

[3] Haynes R., Zhu D., Judge P. K., Herrington W. G., Kalra P. A., Baigent C. (2020). Chronic kidney disease, heart failure and neprilysin inhibition. *Nephrology Dialysis Transplantation*.

[4] Horodinschi R. N., Bratu O. G., Dediu G. N., Pantea Stoian A., Motofei I., Diaconu C. C. (2020). Heart failure and chronic obstructive pulmonary disease: a review. *Acta Cardiologica*.

[5] Jones N. R., Roalfe A. K., Adoki I., Hobbs F. R., Taylor C. J. (2019). Survival of patients with chronic heart failure in the community: a systematic review and meta-analysis. *European Journal of Heart Failure*.

[6] Berglund F., Piña P., Herrera C. J. (2020). Right ventricle in heart failure with preserved ejection fraction. *Heart*.

[7] Zhao B., Sun S., Wang Y. (2021). Cardiac indicator CK-MB might be a predictive marker for severity and organ failure development of acute pancreatitis. *Annals of Translational Medicine*.

[8] Wang S., Li M., Wang X. (2021). The ratio of NT-proBNP to CysC1.53 predicts heart failure in patients with chronic kidney disease. *Frontiers in Cardiovascular Medicine*.

[9] Wang Y., Xu Z., Zhou Y. (2021). Leukocyte cell population data from the blood cell analyzer as a predictive marker for severity of acute pancreatitis. *Journal of Clinical Laboratory Analysis*.

[10] Altay H. (2021). Hyperkalemia in chronic heart failure. *Turk Kardiyoloji Dernegi Arsivi-Archives of the Turkish Society of Cardiology*.

[11] Książczyk M., Lelonek M. (2020). Angiotensin receptor/neprilysin inhibitor-a breakthrough in chronic heart failure therapy: summary of subanalysis on PARADIGM-HF trial findings. *Heart Failure Reviews*.

[12] Dewan P., Docherty K. F., Bengtsson O. (2021). Effects of dapagliflozin in heart failure with reduced ejection fraction and chronic obstructive pulmonary disease: an analysis of DAPA-HF. *European Journal of Heart Failure*.

[13] Mesquita T., Lin Y. N., Ibrahim A. (2021). Chronic low‐grade inflammation in heart failure with preserved ejection fraction. *Aging Cell*.

[14] Wei H., Zhang J., Tang Q. (2017). MiR-638 inhibits cervical cancer metastasis through Wnt/*β*-catenin signaling pathway and correlates with prognosis of cervical cancer patients. *European Review for Medical and Pharmacological Sciences*.

[15] Cardinale D., Colombo A., Bacchiani G. (2015). Early detection of anthracycline cardiotoxicity and improvement with heart failure therapy. *Circulation*.

[16] Chaitman B. R., Alexander K. P., Cyr D. D. (2021). Myocardial infarction in the ISCHEMIA trial: impact of different definitions on incidence, prognosis, and treatment comparisons. *Circulation*.

[17] Charokopos A., Griffin M., Rao V. S. (2019). Serum and urine Albumin and response to loop diuretics in heart failure. *Clinical Journal of the American Society of Nephrology*.

[18] El Iskandarani M., El Kurdi B., Murtaza G., Paul T. K., Refaat M. M. (2021). Prognostic role of Albumin level in heart failure: a systematic review and meta-analysis. *Medicine*.

[19] Jang S., Yang D., Kim H. (2020). Prognostic value of Cystatin C-derived estimated glomerular filtration rate in patients with acute heart failure. *Cardiorenal Medicine*.

